# Sarcopenia modelling by portal vein ligation inducing hyperammonemia in rats

**DOI:** 10.1371/journal.pone.0337178

**Published:** 2025-11-21

**Authors:** Maria Nadinskaia, Kseniya Gulyaeva, Aleksandr Sukhinin, Alla Sedova, Polina Boykova, Ilya Izmailov, Ksenia Pokidova, Egor Kuzmin, Artem Venediktov, Igor Meglinski, Gennadii Piavchenko

**Affiliations:** 1 Department of Internal Medicine, Gastroenterology, and Hepatology, I.M. Sechenov First Moscow State Medical University (Sechenov University), Moscow, Russia; 2 Hand Microsurgery Center, Clinical Hospital named after A.K. Eramishantseva, Moscow, Russia; 3 Department of Human Anatomy and Histology, I.M. Sechenov First Moscow State Medical University (Sechenov University), Moscow, Russia; 4 College of Engineering and Physical Sciences, Aston University, Birmingham, United Kingdom; Mazandaran University of Medical Sciences, IRAN, ISLAMIC REPUBLIC OF

## Abstract

Sarcopenia is a progressive muscle wasting condition often associated with hyperammonemia. However, no approved animal models of sarcopenia with hyperammonemia were reported. This study aimed to provide a surgical modelling of sarcopenia with hyperammonemia. Male Wistar rats were assigned by the method of random numbers (*n* = 6 per group) into experimental group with ligation of portal and pyloric veins or control group with sham surgery. Blood ammonia levels were measured directly after the surgery (20 min), after 1 h to observe acute damage in functioning shunts, and at the final endpoint (30 days). Rats were sacrificed with histological study of the liver, spleen, cerebral cortex, and skeletal muscles. Experimental rats revealed hyperammonemia at 30 days compared to controls, 70 µmol/L versus 38 µmol/L, p <0.05. No significant changes were observed in liver morphology between the groups, approving hyperammonemia without liver damage. Splenomegaly and Gamna-Gandy bodies in the spleen of experimental rats indirectly evidenced functionable portosystemic shunting after the ligation. Cerebral cortex showed a significant decrease in neurons of experimental animals, 7.6 ± 2.5 NeuN^+^cells vs 13 ± 2 in controls, p <0.05. Skeletal muscles revealed a significant difference of muscle fiber diameter between the groups, 20.2 ± 2.1 µm in the experimental group vs 30.7 ± 4.3 µm in controls, at p < 0.001. A model of sarcopenia with hyperammonemia was established with concomitant changes in cerebral histology revealed. This model may be a valuable tool for studies of sarcopenia and related therapeutic options.

## Introduction

Sarcopenia is a muscle failure with multiple adverse changes that accrue across a lifetime, as stated by the consensus at the 2^nd^ session of European Working Group on Sarcopenia in Older People in 2018 [1]. Referred to as an age-related loss of muscle mass since 1989 [2], the term’s meaning was later expanded to include a decline in muscle strength and function of polyfactorial origin with an increased risk of unfavorable clinical outcomes [3]. The clinical significance of sarcopenia requires a development of its relevant models in animals [4].

Nowadays, sarcopenia is often regarded in relation to age-independent factors (e.g., chronic liver disease) [5]. Recent meta-analyses have reported sarcopenia to manifest in almost one third to one half of patients with liver cirrhosis [3,6–8] thereby worsening their quality of life [9], as well as increasing length of hospital stay [10] and mortality rate [11]. The prevalence however varies widely that perhaps may be explained by a large difference in regional alimentary habits, degree of addictions such as alcohol consumption, and overall access to medical care that together change the mode of liver disease course (e.g., by direct ethanol or its metabolites action on skeletal muscles) [12–15].

In liver cirrhosis, the pathogenesis of sarcopenia comprises several interrelated factors, and hyperammonemia is crucial among them [16,17]. Cirrhotic patients develop hyperammonemia due to the portosystemic blood shunting and a decreased liver potential to detoxify gut-originated ammonia [18,19]. Indeed, hyperammonemia enhances proteolysis and autophagy, at the same time suppressing protein synthesis in muscles [20,21] via myostatin signaling and phosphorylation of eukaryotic translation initiation factor 2α, as well as diminished α-ketoglutarate and leucine levels [19,22]. Therefore, chronic hyperammonemia stimulation can be an adequate approach for sarcopenia modelling.

Hepatotoxic medications and/or pollutants, such as acetaminophen or chlorpyrifos, are common to provoke a decrease in ammonia detoxification by a direct damage of hepatocyte productivity [23,24]. For instance, models of toxic liver damage with sarcopenia development in mice and rats have been reported [25,26]. Nevertheless, these studies had no approved increase of blood ammonia. Besides, portal vein surgery can be used to induce hyperammonemia while preserving the liver’s ability to detoxify ammonia. For example, Lattanzi and colleagues showed sarcopenia to accompany portosystemic shunting without liver damage in up to 35% of patients with non-cirrhotic portal hypertension [27], the rate is approximately equal to that in cirrhosis. This model, perhaps the most successful among the previous ones, lacks data on sarcopenic changes in skeletal muscles.

Exactly, our PubMed search has revealed no well-characterized studies of surgical models for portal vein ligation, surgical or spontaneous portosystemic shunting demonstrating sarcopenia with hyperammonemia. Meanwhile, encephalopathy, another common event in hyperammonemia, develops after surgical remodeling of liver blood flow in rats [28,29], rabbits [30], dogs [31], and pigs [32]. Therefore, there is a need for approved models of sarcopenia to obtain a comprehensive set of allowing an evaluation of hyperammonemia effects. Our study aims to develop a model of sarcopenia in rats by portal vein ligation inducing hyperammonemia. We hypothesize whether sarcopenia with hyperammonemia and (considering the number of previous studies for encephalopathy) concomitant encephalopathy can occur in portosystemic shunting without any morphologically demonstrated liver damage.

## Materials and methods

### Animals

We selected male Wistar rats (*n* = 12), 3 month-old and weighing 250–270 g, after a quarantine of 2 weeks. All the animals survived until the end of the study. The rats were randomized by the method of random numbers into two groups (*n* = 6 per group) with stratification criterion of body mass. An experimental group served for sarcopenia modelling, and a control one had a sham surgery. The randomization, surgeries, tissue collection for histological study, and staining were provided by different people to provide blinding and avoid potential bias.

The animals were housed three per cage (no accidents related to animal social behavior were observed during the experiment) with respect to their randomization, at a room temperature of 22–24 °C, relative humidity of 50–70% and 12 h light-dark cycle, with free access to water and standard granulated feeding *ad libitum* in accordance with the principles of Good Laboratory Practice (GLP) and Guide for the Care and Use of Laboratory Animals [33], which is also consistent with local regulatory acts (Russian Federal State Standarts GOST 33044–2014 Principles of good laboratory practice, GOST 33215–2014 Guidelines for accommodation and care of animals. Environment, housing and management, GOST 33216–2014, Guidelines for accommodation and care of animals. Species-specific provisions for laboratory rodents and rabbits). Every day, the animal health and behavior were monitored by a staff trained in animal care and handling. The study design and planned animal mortality are approved by Local Ethical Committee of Federal State Autonomous Educational Institution of Higher Education I.M. Sechenov First Moscow State Medical University of the Ministry of Health of the Russian Federation (Sechenov University), protocol # 20–22 from October 20th, 2022.

### Surgery

Sarcopenia was modeled by ligating the portal vein and its tributary, the pyloric vein, according to a common method [34]. For anesthesia, injections of xylazine at the dose of 2 mg/kg (Interchemie, Netherlands), tiletamine/zolazepam at the dose of 60 mg/kg (Virbac, France) were used with anesthesia depth monitored by a simultaneous dissapear of such reflexes as righting, hind limb withdrawal, and blinking. Perioperative care included the control of respiration rate every 10 min. For ammonia level detection, we inserted a catheter (outer diameter 0.8 mm, inner diameter 0.4 mm; SciCat, Russia) into the left external jugular vein according to a previously reported method [35,36] for blood sampling. The catheter patency and correct placement have been confirmed by drawing 0.1 mL of blood into a discarded syringe then locking with 4% sodium citrate solution.

After the catheterization, we provided surgical access by a layered incision in the upper abdomen along the midline (Fig 1A, B). The small intestine and stomach were examined (Fig 1C, D), and then the portal vein was accessed by the hepatic portal vein isolation at the hepatoduodenal ligament (Fig 1E). We exerted a 10−0 polypropylene suture at the portal trunk before its bifurcation into the lobar veins and at the pyloric vein (Fig 1F, K). For visual post-assessment, we observed early signs of portal hypertension including dilation of the splenic and superior mesenteric veins and venous congestion in the small intestine and stomach (Fig 1G, H). Finally, wound closure was accomplished with a layered suture followed by antiseptic treatment (Fig 1I, J) and by recovery from anesthesia. After the surgery, we injected each rat subcutaneously with 5 ml of saline.

**Fig 1:** Surgery design. **Sarcopenia modeling by ligation of portal and pyloric veins for infrahepatic portal hypertension.** Abbreviations at the figure: L – liver, S – stomach, SI – small intestine, IVC – inferior vena cava, HPV – hepatic portal vein, SMV – superior mesenteric vein, PV – pyloric vein, SV – splenic vein. (A) anesthesia, shaving, marking of the surgical field. (B) access to the abdominal cavity. (C) visual examination of small intestine before the ligation. (D) visual examination of stomach before the ligation. (E) access to the portal vein and its tributaries. (F) surgical area with ligation site. (G) venous congestion in small intestine. (H) venous congestion in stomach. (I) abdominal suture. (J) skin wound closure. (K) illustration of ligation sites.

### Blood ammonia measurement

Blood for ammonia level measurement was sampled at the following time points: on Day 1 from the left external jugular vein immediately before the surgery, 20 min after the ligation, and 1 h after the ligation. On Day 30, ammonia levels were measured in both groups immediately before the sacrification. All the tests were performed at the same time (9–10 am) in standardized fasting state for 3 h to avoid any additional bias from food metabolism.

For the detection, a portable PocketChem BA PA-4140 device, operating on a single-wavelength reflectance (spectrophotometric) method, was employed with disposable reagent test strips of Ammonia Test Kit II (Arkray Factory, Japan). Measurements were performed immediately after sampling, without the use of any conserving media, in order to determine the ammonia concentration in whole blood. The device provides a rapid assessment of minor blood quantities. For the analysis, 20 µL of whole blood in a glass microcapillary was transferred to a test strip. Values for ammonia levels are presented in µmol/L.

### Specimen preparation and histological study

All animals were sacrificed at the same term to provide comparable data for detecting hyperammonemia-related changes, thereby humane endpoints are not applicable. Animals were anesthetized with xylazine at the dose of 2 mg/kg (Interchemie, Netherlands) and tiletamine/zolazepam at the dose of 60 mg/kg (Zoletil-100; Virbac, France) one month after the portal vein ligation, then sacrificed by perfusion of 0.002% heparin solution and *in vivo* fixation in 10% neutral buffered formalin (BioVitrum, Russia). After the perfusion, the brain, liver, spleen, and skeletal muscles (m. rectus abdominis and m. quadriceps femoris) were collected to obtain samples, further fixed in formalin for 48 h (different size of samples, 0.3–0.5 cm, employed to reach optimal preservation quality for this timing) at room temperature. The samples were washed and dehydrated by a standard protocol in isopropanol of increasing concentration, followed by embedding in Histomix Extra paraffin (BioVitrum, Russia). Sections of 3 µm (*n* = 6 per organ sample of each animal) were prepared from paraffin cassettes with a rotary HM325 microtome in accordance with manufacturer’s recommendations (Thermo Fisher Scientific, USA).

Hematoxylin and eosin staining was used to detect changes in the spleen, toluidine blue staining by Nissl served to determine neuronal compartments [37,38], van Gieson’s staining was to reveal connective tissue in the liver [39], and Weigert’s iron hematoxylin staining [40] was intended to show sarcomeres in skeletal muscles (all dyes: BioVitrum, Russia).

Immunohistochemical (IHC) study included a processing with One-step Dewaxing/Antigen Retrieval Buffer (E-IR-R220A, XF05RT4N9592; Elabscience, PRC) at pH of 9, 98 °C, and 105 kPa. The sections were washed three times in phosphate-buffered saline (PBS), incubated with bovine serum albumin (BSA) for 20 min at 37 °C. Rabbit monoclonal antibodies to NeuN (1:50, catalog number ET1602−12, lot H661803001; Huabio, PRC) were employed. After 1.5 h of incubation, the sections were washed with PBS, followed by secondary polyclonal antibodies, conjugated with horseradish peroxidase (Anti-Rabbit-HRP, catalog number HA1119, lot M05-22-P2; Huabio, PRC), and DAB as chromogen. The sections were mounted in xylene-containing Vitrogel medium (HM-VI-A500, 0181, BioVitrum, Russia). The IHC protocol is approved by the manufacturer’s recommendations and reported in studies before as appropriate for samples from rats [41,42]. We also have used two sections (myocardium and hippocampus from a healthy animal) for positive and negative control in each round of IHC study.

Imaging and histological analysis were performed with an Axio Imager.A1 microscope, Axiocam 305 camera, and Zeiss Zen 3.10 software (all elements: Zeiss, Germany). We employed at least 300 dpi resolution and magnification of ×200 (×400 for Van Gieson’s staining). Morphometric analysis was performed using software QuPath 0.5.1 [43], with surface area analysis at ×200 magnification for hemosiderin quantification and 20 muscle fibers measured for muscle fiber diameter. NeuN-positive cells were considered manually per 6 fields of view at different sections per animal as morphologically mature neurons and defined visually as cells with evident DAB expression in both nuclei and perykarya of the neurons. To avoid inter- and intra-observer variability, we performed four rounds of measurements (two by two separate investigators) and considered the data to be credible only after Cohen’s kappa comparison showing more than 0.9 for inter- and intra-observer variability.

### Statistical analysis

Statistics were processed with GraphPad Prizm v10.4.1 (Dotmatics, Boston, MA, USA) and OriginPro 2021 (OriginLab, Northampton, MA, USA). The distribution was assessed with Shapiro-Wilk criterion for histological parameters, as well as with Kolmogorov-Smirnov test and Cramér-von Mises criterion for ammonia levels. Descriptive statistics for normally distributed variables are presented as mean ± standard deviation, while data for otherwise distributed variables are presented as median and interquartile range (25th; 75th percentiles).

For comparison between the control and experimental groups, the Mann-Whitney U-test (for non-Gaussian distribution) and Student’s t-test (for normal distribution) were used in histology, while the Wilcoxon test (to compare data between the groups with respect to the results of Cramér-von Mises testing) and paired Student’s t-test (for within-group time-dependent comparisons) were used in ammonia level measurements, correspondingly. No *post hoc* testing was applicable as there were two groups included in the study.

Differences were considered significant at p < 0.05 and statistical power not less than 0.95 assessed with actual and hypothetical power applications. For inter- and intra-observer variability in IHC study morphometrics, we employed Cohen’s kappa test in cross-tabulation application.

### Sample size estimation

Sample size per animal was calculated on the base of muscle fiber width as key study parameter for two pilot animals included to the groups to satisfy the requirement of minimal but significant animal number possible with respect to 3R principles as following:


$$n=\;\frac{{\text{2}\sigma^{\text{2}}\left(Z\alpha /\text{2}+Z\;\beta \right)}^{\text{2}}}{\delta^{\text{2}}},$$

where “*n”* marks the sample size; “*σ”* – maximal standard deviation; “*Zα”* – target statistical significance level at 1.96 for 95% confidence interval; *“Zβ”* – targeted statistical power (0.8, although 0.95 value of statistical power has been showed for all the experiments); *“δ”* –differences between the groups. The calculations with data from the pilot experiment have provided us with resulting 0.28 animals sufficient for the study, the number enlarged to the minimal common number standard for animal studies and the reproducibility of this model. After the whole study finished, we re-calculated the sample size for each parameter, and these data stayed consistent with pilot ones.

Besides, for each histological parameter, we assessed 6 fields of view from each animal for any staining method. No data were missed throughout the study, so no handling of missed data was required.

## Result

To assess the relevance of the model, blood samples were tested for ammonia concentration (further represented as median and interquartile ranges). In the experimental group, the initial blood ammonia content was 40 µmol/L (33; 43). After the ligation, it increased reaching 52 µmol/L (38; 58) at 20 min, and also 58 µmol/L (53; 88) at 60 min, both different from the initial levels at p <0.05. On Day 30, the ammonia levels remained elevated at 70 µmol/L (59; 81), different from the values of the control group, exactly 38 µmol/L (32; 46), at p <0.05.

Pathological changes in the spleen, such as sclerosis and hemosiderosis, were mild to moderate in the experimental group, and the spleen exhibited multiple hemosiderin deposits (Fig 2A). Morphometric analysis revealed that, on average, 18.9 ± 2.2% of the 100 × 100 µm field of view was occupied by hemosiderin aggregates, p < 0.001 (Fig 2B). Besides, at the macromorphology, spleen of experimental rats stayed larger than of control ones, while a liver atrophy has been seen both visually and according to weight measurement (Fig 3). Meanwhile, no pathological changes were observed in the liver and spleen of the control group when assessed by a common score system [44]. The liver had normal cytoarchitectonics, and the spleen displayed areas of white and red pulp with well-defined nuclei and no sign of hemosiderosis.

**Fig 2:** Morphometric analysis of histological slides in sarcopenia modeling by portal vein ligation and pyloric vein ligation. **(A)** Microphotographs: spleen, hematoxylin and eosin staining, × 200; liver, Van Gieson’s staining, × 400; skeletal muscle, Weigert’s iron hematoxylin staining, × 200; primary motor cerebral cortex (M1, Bregma +0.48 mm), toluidine blue by Nissl, × 200, and antibodies to NeuN, × 200. **(B)** Graph showing the differences in hemosiderin content per 100 × 100 µm field of view. **(C)** Graph showing the differences in muscle fiber width in micrometers. **(D)** Graph showing the differences in the number of NeuN^+^ cells per 100 × 100 µm field of view. *** – p < 0.0001. Arrows mark the pathological changes described in the text.

**Fig 3:** Liver and spleen mass in sarcopenia-hyperammonemia modelling on Day 30. Liver mass (on the left) decreased, while spleen mass (on the right) increased in experimental group after portosystemic shunting with proven hyperammonemia and sarcopenia compared to the control group. *** p <0.001.

Approving hyperammonemia and signs of spleen damage with no severe liver damage, we regarded the model for changes in skeletal muscles. In the experimental group, some areas of hypo-/atrophic changes were revealed, considered as sarcopenia. In the control group, skeletal muscle specimens had a normal structure of sarcomeres, normochromic nuclei, and clearly visible striation. At morphometric analysis, the average muscle fiber width in the control group was 30.7 ± 4.3 µm, compared to 20.2 ± 2.1 µm in the experimental group with the significant difference at p < 0.001 (Fig 2C).

Paying attention to the common testing of encephalopathy in models of chronic liver diseases as shown in introduction, we also studied the specimens of cerebral cortex. In the primary motor cortex, the experimental group had local spongiosis, perineuronal edema, and vacuolated neuronal cytoplasm with some cells staying karyopyknotic, in respect to a common neuropathological scoring system [45]. However, the control group exhibited typical cerebral cytoarchitectonics with intact neurons. Immunohistochemical staining with antibodies to NeuN showed a significant reduction in the number of neurons per 100 × 100 µm field of view in sarcopenia modelling (Fig 2D). The morphometric analysis revealed an average number of 13 ± 2 NeuN^+^ cells in *t* test for the control group comparing to 7.6 ± 2.5 NeuN^+^ cells in the experimental group, the difference is significant at p <0.001.

## Discussion

Multiple studies have demonstrated that sarcopenia worsens the prognosis of severe liver disease with impaired ammonia detoxification, thereby encouraging development and validation of sarcopenia models in hyperammonemia [6,7,14,15,46,47]. Two main approaches are possible to exclude the liver from ammonia detoxification, relying on toxic liver injury [48–50], portocaval shunt surgery [51–53]; or both of them can be combined [54]. This study preferred the surgical approach considering it to avoid potential adverse effects that any medications have. Although Bengtsson et al. and Castaing et al. [51,52], also implemented the approach, sarcopenia was not considered in the Castaing et al. model, and there was insufficient data in the Bengtsson et al. model to postulate hyperammonemia–sarcopenia. Meanwhile, our study has shown a proven combination of sarcopenia by histological analysis and hyperammonemia by biochemical analysis with patency of portosystemic shunting also demonstrated by the presence of Gamna-Gandy bodies in the spleen, as well as splenomegaly and liver atrophy compared to the rats of control group showing the remodeling of portal blood flow.

Comparing experimental and control groups, we found experimental animals to be strongly hyperammonemic, thereby the model tested allowed to provoke hyperammonemia. Indeed, peripheral blood ammonia levels peaked 1 h after the surgery. Further, it stayed elevated by 2-fold until the term of 30 days. Besides, liver histology showed no difference between the groups when assessed by liver disease activity score [44], therefore implementing the concept to avoid additional mechanisms of pathogenesis probable in liver damage.

Meanwhile, histological analysis revealed numerous changes in the spleen, skeletal muscles, and brain of experimental rats. Splenic parenchyma exhibited hemosiderin deposits, Gamna-Gandy bodies, occupying ~19% of visual field (100 × 100 μm). Indeed, portal vein ligation is known to induce acute portal hypertension and splenic venous congestion, which can be morphologically confirmed by the presence of Gamna-Gandy bodies. These are splenic parenchymal hemorrhages followed by calcification [55,56].

Moreover, we consider gut-derived ammonia [57], lacking detoxification in the liver, accumulated and resulted in hyperammonemia underlying both cerebral and muscular pathology [58,59]. Study of cerebral cortex with respect to nervous tissue scoring system [45] revealed neuronal damage with both Nissl staining and immunohistochemistry confirming a 2-fold decrease in number of mature, NeuN-expressing neurons comparing to the controls. Besides, experimental group had spongiosis, perineuronal edema, and vacuolated neuronal cytoplasm with some karyopyknotic cells. Cerebral pathology in hyperammonemia is related to ammonia-dependent activating of NMDA receptors, triggering neuronal death [60]. Key ammonia detoxification pathway in the brain involves astrocytic NF-κB activation and glutamine synthesis with further excitotoxicity and increasing neuronal death [61,62]. Besides, hyperammonemia increases blood brain barrier permeability [63], probably contributing to a higher rate of cortical damage.

Meeting thereby the pre-required conditions (cerebral damage together with no liver morphology affected and hyperammonemia approved), our model also showed sarcopenic changes in skeletal muscles. Skeletal muscles of experimental animals demonstrated pathological changes compared to controls. Increased connective tissue volume and reduced diameter of muscle fiber were observed. Previously, hyperammonemia was reported to result in mitochondrial dysfunction and oxidative stress in skeletal muscle [64] with myostatin upregulation via NF-κB pathway [65].

In our study, a model of sarcopenia in hyperammonemia has been established and characterized. The surgical access demonstrated its relevance, also mentioned by literature as easily feasible [51] and correctable [66]. However, numerous versions of surgical procedures are possible for portal vein ligation [67], and the further usage of this model requires a widened design with their testing, as the implications of this variability might affect reproducibility and translatability.

Concomitant cerebral damage in this model is a valuable finding, as blood ammonia can be detoxified not in the liver only, and portal vein ligation does not automatically mean a neuronal damage in many cases [68]. Scorticati and colleagues reported that isolated portal vein ligation lacked efficiency for cerebral damage modelling without additional toxic injury [69], so our data provide a novel insight into this well-known problem. However, we assume that the isolated portal vein ligation model described by Scorticati was only partially suitable modelling cerebral changes, since the animals were sacrificed too early (on Day 14) to allow behavioral alterations to appear.

Sarcopenia pathophysiology requires further elucidation (Fig 4) but our model provides a platform for further studies of sarcopenia and developing therapeutic strategies for sarcopenic patients. For instance, a medication testing in models with hyperammonemia and cerebral damage for liver cirrhosis [70,71] may become more accurate when compared with testing at hyperammonemia with encephalopathy and sarcopenia but without liver damage. Moreover, there is a growing body of evidence for hyperammonemia occurring in patients without liver damage at all [72–74], and that makes our model even more relevant.

**Fig 4:** Pathophysiological mechanisms linking hyperammonemia to sarcopenia and cerebral changes. On the left: liver (at the center) detoxifies ammonia brought from the gut to remove it as urea in the kidneys further. In portal vein occlusion or in liver pathology, the detoxification lacks efficiency, so numerous effects of hyperammonemia can be observed in skeletal muscles, brain, and spleen. On the right, the structural and molecular outcomes of these effects in skeletal muscles are briefly showed resulting in mitochondrial dysfunction and myostatin upregulation. Abbreviations at the figure: ERK 1/2 – extracellular signal-regulated kinase 1/2; IKK – IκB kinase; mTORC1 – mammalian target of rapamycin complex 1; RHGB – Rh family, B glycoprotein (ammonia transporter); ROS – reactive oxygen species; TAK1 – transforming growth factor β activated kinase; TRAF6 – tumor necrosis factor receptor associated factor 6.

Besides, studies are required for gut microbiota affecting the hyperammonemia-related conditions [75], and our model is actual for the case. For instance, microbiota-related effects via ammonia levels are involved in numerous pathologies in elderly people, and a lot of clinical studies concerning the problem launch every year, all requiring pre-clinical models of sarcopenia-hyperammonemia testing [76].

Other intestine-related factors may induce sarcopenic changes even in normal ammonia level due to the secondary effects of portal hypertension (i.e., intestinal malabsorption and inflammation). A decreased production of short-chain fatty acids by intestinal bacteria, which can affect the synthesis of muscle fibers, may decrease, as well as an imbalance between bacteria producing pro- and anti-inflammatory cytokines also leads to a damaging catabolic impact on muscle fibers [77–79].

### Study limitations and perspectives

1. The number of animals for the sarcopenia modeling was limited due to the ethical reasons and 3R principles, although stayed sufficient considering the statistical calculations.
2. A calibration of the model should consider a longer study duration. In our study, we designed a proof-of-concept model that has not required a larger timing.
3. Only blood ammonia levels and morphological parameters were tested. To verify the efficiency of portosystemic shunting and altered circulation, one may assume computed tomography and/or measurement of manganese levels in the peripheral blood in future studies, as well as measuring portal pressure using a pressure gauge and the degree of bypass using colored polystyrene microspheres. Besides, additional methods of blood ammonia testing can be appropriate for a larger accuracy (enzymatic assay using glutamate dehydrogenase). Promising testing options may include electrophysiological and motor physiological tests (grip strength test, treadmill endurance) to provide a functional correlation to structural changes, dual-energy X-ray absorptiometry and measuring of serum markers levels (e.g., myostatin, creatine kinase, cytokines, atrogin-1, ubiquitin E3 ligases such as muscle RING-finger protein-1) to strengthen mechanistic insights, and molecular approaches (such as blotting and quantitative polymerase chain reaction for detection the relevant proteins and their mRNA, correspondingly, in cell cultures, as well as detection kits for mitochondrial enzymes and their activity are applicable to assess the cell metabolism).
4. Reversibility of sarcopenic changes in this model should be further regarded with hypoammonemic agents. For instance, the usage of rifaximin and L-ornithine-L-aspartate can be appropriate [80].

## Conclusions

Our work proposed an approach of hyperammonemia induction by portal vein ligation. This model of surgical damage was approved to provoke sarcopenia in the absence of liver damage, but with alteration of the brain and spleen. Thus, we developed a model of sarcopenia in rats by portal vein ligation with hyperammonemia. Previous literature references from PubMed database do not describe such a model earlier that is both easy-to-do and appropriate for no liver damage. The model can be a promising tool for studies of hypoammonemic therapies, as well as of sarcopenia-associated diseases.

## Supporting information

S1 File Supporting information – data for plots. This file provides the numerical data from the experimental study. Sheet “Blood ammonia” includes data on ammonia measurement with post hoc sample size re-estimation with respect to these results. Sheet “Mass or organs” represents data on weighing the liver and spleen immediately after the animal sacrification with post hoc sample size re-estimation for this parameter. Sheet “Morphometric values” shows the means of numerical data for the records of cell count in morphometric study at histological slides of skeletal muscles, spleen, and cerebral cortex. Sheet “Pilot, sample size estimation” provides details about initial calculations for primary definition of the sample size.
(XLSX)
